# Peptide ARHGEF9 Inhibits Glioma Progression via PI3K/AKT/mTOR Pathway

**DOI:** 10.1155/2023/7146589

**Published:** 2023-02-18

**Authors:** Jie Huang, Xiaoling Fu, Qiang Xue, Peng Ma, Yating Yin, Minjie Jiang, Yunpeng Lu, Qi Ying, Jun Jiang, Hua He, Da Wu

**Affiliations:** ^1^Department of Neurosurgery, Third Affiliated Hospital, Navy Medical University, Shanghai, China 200432; ^2^Department of Medical Psychology, The Fourth Medical Center of PLA General Hospital, 51 Fu Cheng Road, Beijing, China 100048; ^3^Department of Neurosurgery, Yixing People's Hospital, Yixing, Jiangsu Province, China 214200; ^4^Endoscopy Center, Minhang Hospital, Fudan University, Shanghai, China

## Abstract

**Background:**

The most prevalent malignant tumor in a human brain nervous system is called glioma. Peptide is a compound formed by the peptide bond of *α*-amino acids, and the development of polypeptide drugs has been widely used in many fields. We plan to investigate the underlying peptides with clinical value in glioma.

**Method:**

Based on public databases, we targeted the common genes between glioma differentially expressed genes (DEGs) and peptide genes related to glioma prognosis. Then, these common genes were analyzed by LASSO-Cox analysis, prognostic risk model, and nomogram to identify key prognostic peptide genes and the target gene in this study. Next, the mechanism of target gene in glioma was explored by bioinformatics analysis and functional experiments.

**Results:**

We obtained a total of 26 overlapping genes for the following study. After that, 6 independent prognostic factors (REPIN1, PSD3, RDX, CDK4, FANCI, and ARHGEF9) were obtained and applied to construct the prognostic nomogram, and ARHGEF9 was the target gene in the study. Next, peptide ARHGEF9 was found to inhibit glioma cell development. Through Spearman's correlation analysis, ARHGEF9 had a close relation with PI3K/AKT/mTOR pathway. In functional experiments, peptide ARHGEF9 could suppress the protein expressions of p-PIK3K, p-AKT and p-mTOR, while IGF-1 could reverse this effect.

**Conclusion:**

This study identifies 6 new prognostic biomarkers for glioma patients. Among them, peptide ARHGEF9 gene is an inhibitory gene functioning by targeting PI3K/AKT/mTOR pathway.

## 1. Introduction

Gliomas are the brain and spinal cord tumors originating from glial cells featured with a low 5-year overall survival (OS) and a high mortality [1, 2]. At present, imaging examination is widely applied in disease diagnosis and the evaluation of postoperative efficacy [3]. Nevertheless, it is easily disturbed by radiation damage and surgery, resulting in poor specificity [4, 5]. Meanwhile, due to the lack of specific examination indicators, the realization of timely diagnosis and therapy is not easy in glioma. Surgical resection, chemotherapy and radiotherapy are important therapies for glioma patients [6]. Since most gliomas expand during aggressive growth, resulting in an unclear boundary between the tumor and normal brain tissues, and the glioma cells infiltrate the brain and migrate from the tumor [7]. Thus, it is very difficult to completely remove the tumor by surgery. Currently, it is still critical to identify sensitive and specific biomarkers for a deep realization of glioma tumorigenesis and glioma patients.

Peptide is an organic compound, formed by dehydration of amino acids, which has a close relationship with protein. Research has demonstrated peptides can effectively affect the body's immune function, enhance immune surveillance, and inhibit cancerous cells in the body [8–10]. Some antitumor peptide drugs have been widely studied and applied in tumor therapy because of their small molecular weight, easy penetration to tumor cells, and antidrug resistance [11, 12]. The literature by Kaewjanthong et al. mention that non-small-cell lung cancer cell growth is inhibited by the expression of the PR-PPD peptide, significantly inhibiting cell growth [13]. Also, NGR peptide could target tumor cells. Mohammadi-Farsani et al. confirm through cellular experiments that *α*-NGR fusion protein effectively inhibits the growth of HT1080 and U937 cancer cells, and has cytotoxic effects on CD13-positive cancer cells [14]. To date, an increasing number of preclinical studies have developed a variety of different peptides with potent abilities in tumor models.

In order to discover pertinent genes in a variety of malignancies in the aspects of molecular diagnosis, pathological categorization, therapy evaluation, prognosis prediction, drug sensitivity, and tumor recurrence, we adopt gene expression profiling [15]. Here, by The Cancer Genome Atlas (TCGA) database, this study is aimed at identifying differentially expressed genes (DEGs) and prognosis-related peptide genes in glioma to find candidate targets and biomarkers for gliomas.

## 2. Materials and Methods

### 2.1. Screening of Glioma DEGs

We obtained all glioblastoma (GBM) and low-grade glioma (LGG) [16] RNAseq data in TCGA. Limma package of R software was applied to study different mRNA expressions. The screening criterion for upregulation was log_2_FC > 1, and downregulation was log_2_FC < −1. Meanwhile, *P* value < 0.5 indicated statistical significance. TCGA [17] database (https://portal.gdc.com) provides gene expression and clinical information on various cancers in patients with multiple stages. Meanwhile, the peptide genes related to glioma prognosis were also acquired from TCGA for the common gene screening.

### 2.2. GO and KEGG Pathway Analysis on Glioma DEGs

Gene Ontology (GO) and Kyoto Encyclopedia of Genes and Genomes (KEGG) are sources for comprehensive gene function analysis and associated high-level genomic functional data. The functional enrichment results of TCGA-DEGs come from the R software package Cluster Profiler, in which color stands for the significance, and the circle size is the enriched genes, and the larger the number, the larger the circle. In the enrichment results, *P* < 0.05 was considered to be enriched in meaningful pathways.

### 2.3. Least Absolute Shrinkage and Selection Operator (LASSO) Regression Analysis

Venn diagrams of prognosis-related peptide genes and glioma DEGs were generated to obtain 26 overlapping peptide genes for the next analysis. Next, 26 overlapping genes were selected for LASSO with ten-fold cross-validation. Glioma patients from TCGA were arranged into the high-risk (*n* = 331) and low-risk groups (*n* = 331) with median risk score as a cutoff. In addition, a Kaplan-Meier survival analysis was applied to contrast the difference in survival. In addition, time-dependent ROC (receiver operating characteristic) analysis was conducted to evaluate the prediction ability. All analyses were conducted using the R language (http://www.r-project.org). Thus, we got 17 significant signature genes for the prognostic value assessment analysis.

### 2.4. Correlation Analysis and Prognostic Nomogram Construction

Two-gene correlation plots of prognostic genes were implemented by the R software package ggstatsplot. Important clinical variables and the above 17 genes were assessed by univariate and multivariate Cox regression methods. Then, nomograms were built using the “rms” package based on multivariate analysis to determine the peptide genes with prognostic value. The calibration curve was applied to compare the predicted and real results. Then, due to previous research and obtained results, peptide ARHGEF9 gene was selected for the further study.

### 2.5. Gene Expression Profiling Interactive Analysis (GEPIA)

Based on 33 tumor samples in TCGA, the expression distribution of ARHGEF9 in tumor and normal samples was validated. Gene Expression Profiling Interactive Analysis (GEPIA; http://gepia.cancer-pku.cn/) offers differential analysis of multiple cancers based on TCGA and Genotype-Tissue Expression (GTEx). We compared ARHGEF9 expression levels in GBM, LGG, and pertinent normal samples using the GEPIA database to determine its roles in gliomas.

### 2.6. Kaplan-Meier Plotter Database

The Kaplan-Meier plotter could analyze the gene expression data and clinical information. To explore ARHGEF9 expressions in LGG and brain tumor total samples, ARHGEF9 was entered into this database. The survival maps included OS, disease-free survival (DFS), progression-free survival (PFS), and disease-specific survival (DSS). Hazard ratios (HR) with log-rank *P* values and 95% confidence intervals were calculated on the webpage. Moreover, Spearman's correlation between ARHGEF9 and pathway scores was analyzed using R software to explore related pathways of ARHGEF9 in glioma.

### 2.7. Cell Preparation

Human astrocytes (NHA) and glioma cells (SW1783, U373) from the Chinese Academy of Sciences were kept in Dulbecco's modified Eagle medium (Gibco, NY) medium with 10% fetal bovine serum (FBS) at 37°C in 5% CO_2_. Then, cells were added 10 *μ*M, 40 *μ*M, 80 *μ*M, and 100 *μ*M of the peptide ARHGEF9 and IGF-1, respectively, for a period of time for subsequent analysis.

### 2.8. Quantitative Polymerase Chain Reaction (q-PCR)

Trizol reagent was adopted to isolate RNA from cells, and then, they were reverse transcribed into complementary DNA by ABI 7500 real-time PCR system (Applied Biosystems, Inc.). q-PCR was then conducted by SYBR Green PCR Master Mix with GAPDH as an internal control. Finally, the results were analyzed by the 2^-*ΔΔ*Ct^ method.

### 2.9. Cell Count Kit-8 Assay

In the cell proliferation viability assay, we firstly added the treated cells to a 96-well plate at a density of 1 × 10^3^. Then, 10 *μ*l of CCK-8 solution was injected into each well plate, and the optical density (OD) values of the cells at 450 nm at 0, 1, 2, 3, and 4 days were calculated using a microplate reader to evaluate the state of cell proliferation.

### 2.10. Transwell Assay

For cell invasion and migration ability, we used the method of Transwell. Tarnswell consists of two chambers, the upper and lower layers, separated by a polycarbonate membrane. The treated cells were first added to the upper chamber of the Transwell with Matrigel, not required for migration assays. After a period of time, the invading and migrating cells were fixed with methanol and stained with crystal violet, and the excess was removed with a cotton swab. Finally, the number of cells invading and migrating in the field of view was observed by microscope, and their invasive and migrating abilities were evaluated.

### 2.11. Statistical Analysis

Statistical analysis was performed using GraphPad Prism 8.0 software and SPSS 20.0 software. All experiments were performed in triplicate. Comparisons between the two groups were made by a paired-samples *t*-test. Three or more experimental groups were compared by one-way ANOVA and post hoc Bonferroni test. All data were presented as the mean ± standard deviation (SD). *P* < 0.05 was considered to indicate a statistically significant difference.

## 3. Results

### 3.1. Identification and Enrichment Analysis of Glioma DEGs

Under adjusted *P* < 0.05 and log_2_FC < −1 criteria, we got 2146 downregulated DEGs, and under log_2_FC > 1, we got 1171 upregulated DEGs (Figure 1(a)). Then, KEGG analysis demonstrated the up-enriched pathways included TGF-beta signaling pathway, p53 signaling pathway, and down-enriched pathways included the cAMP signaling pathway and synaptic vesicle cycle (Figures 1(b) and 1(c)). For GO terms, upregulated DEGs were related to viral transcription and viral gene expression, and downregulated DEGs were enriched in synaptic vesicle exocytosis, vesicle-mediated transport in the synapse, etc. (Figures 1(d) and 1(e)).

### 3.2. Construction and Evaluation of Prognostic Risk Models

Figure 2(a) is a Venn diagram of 196 prognosis-related peptide genes and 3317 DEGs, with 26 overlapping genes. To further identify genes significantly related to glioma prognosis, we performed LASSO regression with ten-fold cross-validation on 26 overlapping genes to obtain the optimal *λ* value from the smallest partial likelihood deviation (*λ*), and finally, 17 prognostic genes were identified (Figures 2(b) and 2(c)). Risk scores were calculated for each patient, where we obtained the median cut-off point using the “survminer” R package.  Figure 2(d) shows the survival status of all patients and the heat map of the 17 prognostic genes. As risk scores increased, patients survived less and died more. KM survival curves demonstrated worse PFS in the high-risk group (Figure 2(e)). Moreover, the prognostic signals of 17 genes indicated larger AUC values in the time-dependent ROC analysis (Figure 2(f)), implying that the risk model had better predictive power in 1-, 3-, and 5-year PFS.

### 3.3. Six Prognostic Peptide Genes Were Identified through a Nomogram

To understand the expression relationship among the 17 prognostic genes, we performed gene correlation analysis (Figure 3(a)). The red dots represented positive correlation and the blue dots negative correlation. Then, we found that REPIN1, PSD3, RDX, CDK4, FANCI, and ARHGEF9 might be independent prognostic variables for gliomas (Figures 3(b) and 3(c)). Next, we designed a composite nomogram with REPIN1, PSD3, RDX, CDK4, FANCI, and ARHGEF9 to predict 1-, 3-, and 5-year OS in glioma patients (Figure 3(d)). From the calibration plot of glioma patient survival prediction, it was evident that the nomogram's prediction findings and the actual outcomes agreed rather well (Figure 3(e)). It was obtained that the above six genes all could be the prognostic biomarkers in gliomas.

### 3.4. Expression Analysis on ARHGEF9 in Pan-Cancers

Figures 4(a)–4(d) show a comparison of ARHGEF9 expression in 33 tumor tissues and normal tissues. We could see that ARHGEF9 was lowly expressed in most tumors, indicating that ARHGEF9 acted as a tumor suppressor gene in most tumors like BLCA (bladder urothelial carcinoma), BRCA (breast invasive carcinoma), COAD (colon adenocarcinoma), and ESCA (esophageal carcinoma).  Figure 4(e) is a boxplot of ARHGEF9 expression in LGG and GBM, which was expressed at a lower level in LGG and GBM tissues. These findings showed that ARHGEF9 functioned as an inhibitory role in glioma.

### 3.5. Survival and Pathway Analysis on ARHGEF9 in Glioma

Next, we conducted a KM survival analysis in glioma patients. OS, PFS, DFS, and DSS with high ARHGEF9 expression in LGG were better than those with low expression (Figures 5(a)–5(d)). In addition, high ARHGEF9 expression indicated higher OS, PFS, DFS, and DSS survival rates in total brain tumor samples (LGG+GBM, Figures 5(e)–5(h)). Moreover, ARHGEF9 was significantly upregulated in the GBM group (Figure 5(i)).

### 3.6. Peptide ARHGEF9 Inhibited the Development of Glioma Cells

We first detected the effects of peptide ARHGEF9 with different concentrations on the proliferation of astrocytes and glioma cells based on the CCK-8 assay. According to the results in Figures 6(a)–6(c), it could be seen that the proliferation of NHA cells was not significantly changed in SW1783 and U373 cells, while the proliferation activity of glioma cells decreased with the increased concentration of peptide ARHGEF9 from 10 *μ*M to 100 *μ*M. In CCK-8 assays, it was observed that peptide ARHGEF9 could block the proliferation of SW1783 and U373 cells (Figures 6(d) and 6(e)). Similarly, in the Transwell experiment, in comparison with the normal control group, peptide ARHGEF9 significantly suppressed the invasion and migration of glioma cells (Figures 6(f)–6(i)). Thus, we concluded that peptide ARHGEF9 inhibited the development of glioma cells.

### 3.7. Peptide ARHGEF9 Downregulated PI3K/AKT/mTOR Signaling Pathway-Related Proteins in Glioma Cells

Next, ARHGEF9 was negatively correlated with 6 pathways in pathway correlation analysis (Figures 7(a)–7(f)), namely, PI3K/AKT/mTOR pathway, EMT markers, DNA repair, tumor inflammation signature, tumor proliferation signature, and apoptosis. Considering that the PI3K/AKT/mTOR signaling pathway showed a close relation with ARHGEF9, we detected the expressions of its related proteins, PIK3K, p-PIK3K, mTOR, p-mTOR, AKT, and p-AKT. In SW1783 and U373 cells after treatment with the peptide ARHGEF9, the expressions of p-PIK3K, p-AKT, and p-mTOR were significantly downregulated compared with the control group (Figures 8(a) and 8(b)). IGF-1, also known as a growth-promoting factor, is a polypeptide protein substance. Herein, we compared the regulation of normal control, peptide ARHGEF9, and IGF-1+peptide ARHGEF9 on glioma cells. In Figures 8(c)–8(f), peptide ARHGEF9 suppressed the proliferation and migration of glioma cells, while IGF-1 could weaken the effect of peptide ARHGEF9 on the proliferation and migration of glioma cells. All in all, these data revealed that peptide ARHGEF9 suppressed glioma by the PI3K/AKT/mTOR signaling pathway.

## 4. Discussion

Gliomas are common primary brain tumors that are rarely curable. Peptides have been applied in clinical practice widely. For instance, it is used as antigen to detect viruses, cells, mycoplasma, and so on [18]. Peptide antigen has strong specificity and is easy for preparation than natural microorganisms or parasites protein antigen [19]. To find biomarkers for glioma, we conducted a series of bioinformatics analyses between glioma and peptide genes. First of all, we identified DEG between glioma and normal samples and glioma-related peptide genes in TCGA database. The overlapping genes were selected to conduct the following analysis for the screening of effective targets or biomarkers.

As for the glioma DEGs, GO term enrichment analysis showed these DEGs were related to functions involving neurotransmitter secretion, neurotransmitter transport, and synapse organization. It is well known that neurotransmitters not only maintain normal brain function but also influence glioma progression. Pei et al. studied the progression of neurotransmitters such as glutamate, calcium, and NO in brain tumors. The results suggested that glutamatergic and calcium signaling might accelerate glioma replication and progression through metabolic reprogramming and gene switching, providing positive feedback to promote glioma formation [20]. Studies by Lin et al. suggest that differentially expressed synapses and synapse-associated proteins (SAPs) may be involved in the formation of glutamate synapses and LGG synapses. Furthermore, they found that SAPs might be related to the pathogenesis of seizures in glioma patients [21]. KEGG pathway analysis indicated the functions of DEGs were mainly concentrated in the Notch, Hippo, and cAMP signaling pathways. Javed et al. showed that the Notch signaling pathway was an evolutionary-conserved pathway affecting the differentiation process from the early embryonic stage to the mature brain [22]. Growing evidence implicates the Hippo pathway in tumor progression and resistance to therapy. Masliantsev et al. suggest the Hippo pathway is connected with the pathophysiology of gliomas [23]. The findings of Jiang et al. suggest FAK/Akt and cAMP/PKA pathways are associated with the process of MOB2 inhibiting GBM [24].

After a series of analyses, we found REPIN1, PSD3, RDX, CDK4, FANCI, and ARHGEF9 might be used as independent prognostic factors. To confirm the prognostic predictive ability of genes, an accurately predictive nomogram of glioma prognosis was designed by REPIN1, PSD3, RDX, CDK4, FANCI, and ARHGEF9. The results demonstrated that they were validated as independent prognostic factors in glioma patients to predict 1-, 3-, and 5-year OS probabilities in patients. In gliomas, a very perfect agreement between predicted and actual outcomes was observed in the calibration plots of our nomograms. This confirms the nomogram can offer treatment guidance and predict the prognosis for glioma patients. Furthermore, based on the implications of our study for the significant clinical significance of prognostic genes, we believe that we provide the need for follow-up functional experimental exploration. Besides, the above six genes have been reported before in other cancers [25–27], while few are about ARHGEF9, so it was determined as the target gene for the next study among the 6 genes.

ARHGEF9 (Cdc42 Guanine Nucleotide Exchange Factor 9) encodes an important neuronal synaptic protein, and loss of ARHGEF9 leads to severe intellectual disability, epilepsy [28], and specific facial deformities which are focused by most researchers. For example, studies by Alber et al. show that ARHGEF9 mutations can cause a motor developmental delay in children or be combined with seizures [28]. The main clinical phenotypes in children with variants in the ARHGEF9 gene include developmental delay, epileptic encephalopathy, and autism spectrum disorder. The findings of Yang et al. suggest seizures are controlled by levetiracetam and valproic acid in children with an epileptic phenotype led by variants in the ARHGEF9 gene [29]. In our study, ARHGEF9 was under expressed in most cancers, including gliomas. For example, Ma et al. showed that ARHGEF9 functions as a tumor suppressor in gastric cancer [30]. Furthermore, low expression of ARHGEF9 led to a poor survival in LGG and GBM patients. In cell experiments, we first treated glioma cells by using different concentrations of ARHGEF9. Compared with normal cells, it was found that the higher the concentration of ARHGEF9, the more obvious the inhibitory effect on the proliferation of glioma cells and also significantly inhibited their ability to invade and migrate. It indicates that peptide ARHGEF9 is a suppressor gene in glioma.

Subsequent Spearman's correlation analysis of ARHGEF9 and pathways showed that 6 pathways were closely associated with ARHGEF9, namely, PI3K/AKT/mTOR pathway, EMT markers, DNA repair, tumor inflammatory signature, tumor proliferation signature, and apoptosis. Studies have confirmed that the PI3K/Akt/mTOR pathway is intimately connected to the growth, metabolism, autophagy process, and treatment resistance of glioblastoma [31, 32]. Yao et al.'s experiments demonstrated that miR-15a and miR-92a can inhibit the development of glioma cells through the PI3K/AKT/mTOR signaling pathway [33]. The role of DNA repair mechanisms leads to drug resistance and tumor recurrence, reducing the efficacy of glioma therapy [34]. In addition, other studies have also shown that tumor inflammation and apoptosis are also related to the occurrence and development of gliomas [35, 36]. Among them, we selected the PI3K/AKT/mTOR pathway with the strongest correlation for the subsequent experimental analysis. Subsequently, we investigated the levels of 6 proteins connected with the PI3K/AKT/mTOR pathway in ARHGEF9-treated glioma cells and discovered the levels of p-PIK3K, p-AKT, and p-mTOR were significantly downregulated. Finally, we evaluated the effect of IGF-1 on glioma cells and found that IGF-1 could reverse the proliferation and migration of ARHGEF9 on tumor cells. All of these results showed the PI3K/AKT/mTOR pathway was related to the mechanism of ARHGEF9 in glioma.

Compared with other similar studies, this study is the first one to explore the function and exact mechanism of peptide ARHGEF9 gene in gliomas. However, this study on the role of ARHGEF9 in glioma cells still has some limitations. The current experiments were all done at the cellular level, and the animal experiments should be further considered in future studies to confirm the current findings.

## 5. Conclusion

Taken together, our results provide evidence supporting that ARHGEF9 functions as a tumor suppressor and prognostic biomarker in gliomas. In addition, *in vitro* experiments confirm that ARHGEF9 could hinder the development of glioma cells and downregulate the levels of PI3K/AKT/mTOR pathway-related proteins. Thus, it is concluded that ARHGEF9 is a glioma suppressor gene that acts through the PI3K/AKT/mTOR pathway, which reveals part of the mechanism between peptides and gliomas and provides a new potential therapeutic target and a prognostic biomarker for patients.

## Figures and Tables

**Figure 1:** Identification of glioma DEGs. (a) Heat map of cluster distribution of DEGs in glioma tissue and normal tissue. (b–e) KEGG pathways and GO terms on upregulated and downregulated DEGs.

**Figure 2:** Construction and evaluation of prognostic risk models. (a) Venn diagram of prognosis-related peptide genes and DEGs. (b) Distribution plot of LASSO coefficients for 26 overlapping genes. (c) Partial likelihood bias of variables. (d) Risk score model and distribution map of survival time in glioma patients. (e) Kaplan-Meier curves of risk scores in glioma. (f) ROC curve analysis.

**Figure 3:** Correlation analysis and nomogram construction. (a) Spearman's correlation analysis among 17 gene expressions. (b) Univariate analysis of 17 genes and clinical characteristics. (c) Multivariate analysis of 17 genes and clinical characteristics. (d) Nomogram of prognostic genes in glioma. (e) Calibration curve.

**Figure 4:** Expression analysis on ARHGEF9 in pan-cancers. (a–d) Expression distribution of ARHGEF9 in 33 tumors. ^∗^*P* < 0.05,  ^∗∗^*P* < 0.01, and^∗∗∗^*P* < 0.001.

**Figure 5:** Prognostic analysis of ARHGEF9 in glioma. (a–d) Probabilistic analysis of OS, PFS, DFS, and DSS of different ARHGEF9 expression in LGG. (e–h) Probabilistic analysis of OS, PFS, DFS, and DSS of ARHGEF9 expression in total glioma samples (LGG+GMB). (i) Comparison of ARHGEF9 expressions in GBM and LGG. ^∗^*P* < 0.05.

**Figure 6:** Peptide ARHGEF9 inhibited proliferation, invasion, and migration of glioma cells. (a) The effect of peptide ARHGEF9 with different concentrations on NHA cells. (b, c) The effect of peptide ARHGEF9 with different concentrations on the proliferation of SW1783 and U373 cells. (d, e) The effect of peptide ARHGEF9 on the invasion of SW1783 cells; the left side is the observed field of view, and the right side is the visual bar graph. (f–i) The effect of peptide ARHGEF9 on the migration of U373 cells; the left side is the observed field of view, and the right side is the visual bar graph. ^∗^*P* < 0.05 and^∗∗^*P* < 0.01.

**Figure 7:** Spearman's correlation analysis between ARHGEF9 and pathway scores. (a) PI3K/AKT/mTOR signaling pathway. (b) EMT marker genes. (c) DNA damage repair. (d) Tumor inflammatory signatures. (e) Tumor proliferation characteristics. (f) Apoptosis.

**Figure 8:** Peptide ARHGEF9 downregulated the expression of PI3K/AKT/mTOR signaling pathway-related proteins in glioma cells. (a, b) The effect of peptide ARHGEF9 on PI3K/AKT/mTOR signaling pathway-related proteins in SW1783 and U373 cell. (c, d) CCK-8 detected the proliferation ability of SW1783 and U373 cells treated with peptides ARHGEF9 and IGF-1. (e, f) Transwell assay detected the migration of glioma cells after treatment with peptides ARHGEF9 and IGF-1. ^∗^*P* < 0.05 and^∗∗^*P* < 0.01, compared with the control group. ^#^*P* < 0.05 and^##^*P* < 0.01, compared with the ARHGEF9 group.

## Data Availability

The datasets used and/or analyzed during the current study are available from the corresponding authors on reasonable request.
